# Fahr Disease: A Rare Cause of First-Time Seizure in the Emergency Department

This article has been retracted.

**DOI:** 10.7759/cureus.19965

**Published:** 2021-11-28

**Authors:** Faleh M Aldawsari, Turki B Alotaibi, Omran S Hashim, Zainab A Bu Hamad, Maha R Eisaa, Abdulrahman A Alhumaidi, Salem M Alanazi, Fahad F Alenezi, Afnan A Batwie, Abdulaziz A Habib, Sukainah S Alismail, Omar S Almulhim, Abdullah F Al Amer, Thamer A Alghamdi, Faisal Al-Hawaj

**Affiliations:** 1 General Practice, ​King Khalid Hospital, Al-Kharj, SAU; 2 Medicine, University of Debrecen, Debrecen, HUN; 3 National Guard Health Affairs, Prince Mohammed Bin Abdulaziz Hospital, Medina, SAU; 4 Medicine, Medical University of Warsaw, Warsaw, POL; 5 Medicine, Sulaiman Al Rajhi University, Qassim, SAU; 6 Medicine, King Saud bin Abdulaziz University for Health Sciences, Riyadh, SAU; 7 Medicine, University of Jordan, Amman, JOR; 8 Medicine, Jordan University of Science and Technology, Irbid, JOR; 9 Medicine, King Abdulaziz University, Jeddah, SAU; 10 General Practice, King Faisal Hospital, Al-Ahsa, SAU; 11 Medicine, King Faisal University, Hofuf, SAU; 12 Medicine, Gulf Medical University, Ajman, ARE; 13 Medicine, Al-Baha University, Al Baha, SAU; 14 Medicine, Imam Abdulrahman Bin Faisal University, Dammam, SAU

**Keywords:** case report, computed tomography, seizure, neuropsychiatry symptoms, fahr disease

## Abstract

Seizure is a common neurological problem in the emergency department. First-time seizure needs careful evaluation to exclude the underlying structural brain lesions. Neuroimaging studies, including magnetic resonance imaging and computed tomography scan, are strongly recommended for all adult patients with first-time seizures. We report the case of a 35-year-old woman who was brought to the emergency department because of the first-time loss of consciousness episode. She developed bilateral jerky movements in both her upper and lower limbs. It was associated with frothy secretions from the mouth and cyanosis. The episode lasted for two minutes and terminated spontaneously. The patient was tired after gaining consciousness. The past medical history of the patient was remarkable for anxiety, depression, and polycystic ovarian syndrome. She has undergone multiple cognitive behavioral therapy sessions, but she did not take any psychiatric medications. Neurological examination did not reveal any focal neurological deficit. The patient underwent a computed tomography scan to exclude any space-occupying lesion. The unenhanced scan demonstrated bilateral symmetrical calcification of the basal ganglia. No calcification was noted in the cerebellum or the cerebral cortex. Otherwise, no intracranial pathology was seen. Such findings conferred the diagnosis of Fahr disease. The patient was discharged on carbamazepine to prevent further seizure episodes. After six months of follow-up, the patient did not experience further convulsion episodes. Fahr disease is a rare disorder with a wide spectrum of manifestations. Despite its rarity, physicians should keep this condition as a possible differential diagnosis when they encounter an adult patient with a first-time seizure, particularly in a patient with a history of neuropsychiatric disorders.

## Introduction

Seizure is a common neurological problem that has a lifetime prevalence of up to 10%. It accounts for 2% of all visits to the emergency department [1]. There are several possible causes of seizures depending on the setting and the type of seizure. Notably, first-time seizures constitute 25% of all seizure cases presenting to the emergency department [2]. In contrast to children, the first seizure in adults is more likely to have an underlying cause. Such patients should be evaluated carefully by an experienced physician because of the broad differential diagnoses of seizures. For example, the primary conditions that need to be considered include syncope, migraine, panic attack, and transient ischemic attack. The evaluation starts with detailed history taking about the seizure episode and assessing for possible risk factors and relevant medical history [3]. Imaging studies are strongly recommended for all adults with first-time seizures. Magnetic resonance imaging is recommended because of its high sensitivity for detecting structural brain abnormalities. However, computed tomography can be used in the emergency setting [2]. Here, we report the case of a first-time seizure in a young woman who was found to have Fahr disease, a rare neurological disorder.

## Case presentation

We present the case of a 35-year-old woman who was brought to the emergency department by her spouse because she developed convulsion for the first time in her life. He reported that while the patient was having her breakfast, she experienced unusual visual and sensory sensations with tinnitus. She was not complaining of any pain or feeling abnormal heartbeats. Suddenly, the patient lost consciousness and fell to the ground. She was not aware of the surrounding. The patient had frothy secretions from the mouth, and her color turned blue. She had repetitive jerky movements of her upper and lower limbs. This episode lasted for two minutes and was terminated spontaneously. After that, the patient regained consciousness, but she was very tired and fell asleep. There was no history of difficulty in speech or weakness following the episode. She did not remember the event. There was no history of early morning headache, nausea, or vomiting.

The past medical history of the patient was remarkable for primary infertility due to polycystic ovarian syndrome for which the patient is on metformin 500 mg daily. She had a long-standing history of depression and anxiety for which she underwent frequent cognitive behavioral therapy sessions. She underwent elective laparoscopic cholecystectomy for recurrent episodes of biliary colic. The patient was a non-smoker and never consumed alcohol. She worked as a lecturer and research assistant. Her family history was significant for breast cancer and Parkinson's disease.

Upon examination, the patient appeared tired. Her vital signs were within the normal limits. She had a heart rate of 90 bpm, respiratory rate of 14 bpm, temperature of 36.8℃, and maintained blood pressure. She was oriented to place, time, and person. There were no speech abnormalities. Neurological examination of the upper and lower limbs showed normal muscle tone and power. The reflexes were normal. She had a normal gait and coordination. Examination of other systems was unremarkable. Further, the initial laboratory investigations revealed no abnormalities (Table 1).

**Table 1:** Summary of the results of laboratory findings

Laboratory Investigation	Unit	Result	Reference Range
Hemoglobin	g/dL	14.1	13.0–18.0
Leukocytes	1000/mL	10.9	4.0–11.0
Platelet	1000/mL	382	140–450
Erythrocyte sedimentation rate	mm/h	14	0–20
C-reactive protein	mg/dL	508	0.3–10.0
Total bilirubin	mg/dL	0.8	0.2–1.2
Albumin	g/dL	3.9	3.4–5.0
Alkaline phosphatase	U/L	55	46–116
Gamma-glutamyltransferase	U/L	16	15–85
Alanine transferase	U/L	18	14–63
Aspartate transferase	U/L	20	15–37
Blood urea nitrogen	mg/dL	10	7–18
Creatinine	mg/dL	0.9	0.7–1.3
Sodium	mEq/L	139	136–145
Potassium	mEq/L	3.9	3.5–5.1
Chloride	mEq/L	104	98–107

Since the patient had no previous history of epilepsy, a computed tomography scan of the head was performed to rule out any space-occupying lesion. The unenhanced scan demonstrated bilateral symmetrical calcification of the basal ganglia. No calcification was noted in the cerebellum or the cerebral cortex. Otherwise, no intracranial pathology was seen. Such findings conferred the diagnosis of Fahr disease (Figure 1). The patient was discharged on carbamazepine to prevent further seizure episodes. After six months of follow-up, the patient did not experience further convulsion episodes.

**Figure 1:** Unenhanced head CT demonstrating bilateral calcification in the basal ganglia CT, Computed tomography.

## Discussion

We reported a case of a first-time seizure in an adult woman who was found to have Fahr disease, which is a very rare neurological disorder characterized by calcification of the basal ganglia. Fahr disease has a population prevalence of less than one case per million [4]. It is named after Karl Theodor Fahr, a German neurologist, who described the first case in 1930. Fahr disease is commonly inherited as an autosomal dominant disorder. However, it may occur sporadically without any family history [5]. Several mutations have been described to be associated with the Fahr disease. Such mutations included the idiopathic basal ganglia calcification-1 (IBGC1) and the solute carrier family 20 member 2 (SLC20A2), which are located on chromosomes 14 and 8, respectively [6]. As in our case, the age of onset of Fahr disease is usually the third and fourth decades.

According to the diagnostic criteria proposed by Moskowitz in 1971 that was later modified by Ellie and Manyam [7], Fahr disease can be diagnosed if there is neuroimaging evidence of bilateral calcification of the basal ganglia with neurologic or neuropsychiatric manifestations. The possible differential diagnoses, including metabolic or mitochondrial disorders, infectious causes, and trauma, need to be excluded. In the present case, the patient fulfilled these criteria.

A computed tomography scan is the preferred neuroimaging study to evaluate the extent of intracranial calcification. Fahr disease typically involves the basal ganglia, especially the globus pallidus, cerebellum, brainstem, and subcortical white matter [7]. In the present case, the calcification was limited to the basal ganglia. The pathogenesis of Fahr disease is not clear. However, it has been associated with endocrine disorders, particularly related to parathyroid glands, dermatological conditions, and infectious diseases [8].

Fahr disease has a wide spectrum of manifestations. It may present with Parkinsonism, tremor, chorea, memory impairment, and poor concentration [7]. While the disease is incurable, the management strategies are targeted toward the relief of symptoms and improving the quality of life of the patient and their caregivers [9].

## Conclusions

Fahr disease is a rare neurological disorder that may have a wide spectrum of manifestations. Despite its rarity, emergency medicine physicians should keep this condition as a possible differential diagnosis when they encounter an adult patient with a first-time seizure, particularly in a patient with a history of neuropsychiatric disorders. A computed tomography scan can provide the neuroimaging evidence of Fahr disease accurately. The treatment strategy should focus on the symptomatic treatment of patients and their quality of life.
